# Quantitative relationship between functionally active telomerase and major telomerase components (hTERT and hTR) in acute leukaemia cells

**DOI:** 10.1038/sj.bjc.6602546

**Published:** 2005-04-12

**Authors:** J H Ohyashiki, H Hisatomi, K Nagao, S Honda, T Takaku, Y Zhang, G Sashida, K Ohyashiki

**Affiliations:** 1 Intractable Immune System Diseases Research Center, Tokyo Medical University, 6-7-1, Nishishinjuku, Shinjuku, Tokyo 160-0023, Japan; 2 Analytical Center for Medical Science, SRL Inc., Tokyo, Japan; 3 Center for Molecular Biology and Cytogenetics, SRL Inc., Tokyo, Japan; 4 First Department of Internal Medicine, Tokyo Medical University, Tokyo, Japan

**Keywords:** telomerase, hTERT, splicing variants, hTR

## Abstract

Functionally active telomerase is affected at various steps including transcriptional and post-transcriptional levels of major telomerase components (hTR and human telomerase reverse transcriptase (hTERT)). We therefore developed a rapid and sensitive method to quantify hTERT and its splicing variants as well as the hTR by a Taqman real-time reverse transcriptase–polymerase chain reaction to determine whether their altered expression may contribute to telomere attrition *in vivo* or not. Fresh leukaemia cells obtained from 38 consecutive patients were used in this study. The enzymatic level of telomerase activity measured by TRAP assay was generally associated with the copy numbers of full-length hTERT+*α*+*β* mRNA (*P*=0.0024), but did not correlate with hTR expression (*P*=0.6753). In spite of high copy numbers of full-length hTERT mRNA, telomerase activity was low in some cases correlating with low copy numbers of hTR, raising the possibility that alteration of the hTR : hTERT ratio may affect functionally active telomerase activity *in vivo*. The spliced nonactive hTERT mRNA tends to be lower in patients with high telomerase activity, suggesting that this epiphenomenon may play some role in telomerase regulation. An understanding of the complexities of telomerase gene regulation in biologically heterogeneous leukaemia cells may offer new therapeutic approaches to the treatment of acute leukaemia.

Human telomerase reverse transcriptase (hTERT) is an essential component of the holoenzyme complex that adds telomeric repeats to the ends of chromosomes (Meyerson *et al*, 1997; Nakamura *et al*, 1997). The differential expression of telomerase in most malignant cells makes it an attractive target for cancer therapy (Mokbel, 2003; Shay and Wright, 2003); however, recent progress in studies on telomerase regulation has shown that telomerase activation is achieved by a process involving various steps including transcriptional and post-transcriptional levels of hTERT gene (Kyo and Inoue, 2002). An alternate splicing of hTERT transcript is one of the regulatory mechanisms of telomerase activity (Ulaner *et al*, 1998). Several alternatively spliced variants of hTERT have been identified (Kilian *et al*, 1997; Ulaner *et al*, 1998; Wick *et al*, 1999; Yi *et al*, 2001); one deletion site induces the *α*-deletion variant, lacking 36 bp from exon 6, and the other induces the *β*-deletion variant, lacking 182 bp from exons 7 and 8 (Yi *et al*, 2001). More recently, we have found a new alternatively spliced form, namely the *γ*-deletion variant, lacking the entire exon 11 (Hisatomi *et al*, 2003; Nagao *et al*, 2004). Since splicing variants are considered to be nonfunctional forms, it is important to discriminate the full-length isoform from variants (Yi *et al*, 2001).

Another essential element to control telomerase activity is the RNA component of telomerase (hTR: human telomerase template RNA) (Feng *et al*, 1995; Weinrich *et al*, 1997). Several lines of evidence suggest the possibility that reprogramming of telomerase by expression of mutant telomerase RNA would result in impaired function of telomeres (Marusic *et al*, 1997). Indeed, germline mutation *hTR* has been found in the autosomal dominant form of congenital dyskeratosis (DKC) showing progressive telomere shortening without functional telomerase activity (Mitchell *et al*, 1999; Vulliamy *et al*, 2001). More recently, it has been shown that heterozygous telomerase RNA mutations found in DKC and aplastic anaemia reduce telomerase activity via haploinsufficiency (Marrone *et al*, 2004).

The aim of this study was therefore to clarify the quantitative relationship between functionally active telomerase and its components hTR and hTERT (and its spliced variants) using a rapid and highly specific real-time quantitative polymerase chain reaction (RT-Q-PCR) and gain greater insight into the complex regulatory system of telomerase in acute leukaemia cells.

## MATERIALS AND METHODS

### Patients and cells

We examined 38 consecutive patients with *de novo* acute leukaemia whose peripheral blood or bone marrow cells contained more than 90% blasts at diagnosis (8–68 years of age): 13 with ALL-L2 and 25 with AML (M1, 6; M2, 14; M3, 2; M4, 2; and M5, 1). *De novo* acute leukaemia was diagnosed according to the French–American–British criteria. All of the ALL patients had precursor B-cell phenotype, and no patient with T-cell ALL was included in this study. Some of the clinical and molecular biological data concerning these patients were reported elsewhere (Ohyashiki *et al*, 2001, 2002). All the samples of peripheral blood or bone marrow cells were separated using a Ficoll–Hypaque gradient, then cell pellets were immediately stored at −80°C. All samples were acquired after obtaining written informed consent from the patients.

### Quantification of telomerase activity

Telomerase activity was assessed by TRAP assay according to the method of Kim *et al* and Piatyszak *et al* with minor modifications, using an automated DNA sequencer (Ohyashiki *et al*, 1997). For standardisation of telomerase activity, we used 10 ag of ITAS/telomerase assay and the level of telomerase activity was arbitrary expressed as the ratio of the TRAP ladder/ITAS per microgram of protein as reported previously (Ohyashiki *et al*, 1997).

### Real-time reverse transcriptase–polymerase chain reaction of hTERT mRNA and hTR RNA

Total RNA was extracted using the RNeasy Mini Kit (Qiagen, MD, USA). Total RNA (1 *μ*g) was used for cDNA synthesis using a Ready-To-Go You-Prime First-Strand Beads (Amersham Biosciences, Piscataway, NJ, USA) and a pd(N)6 Random Hexamer (Amersham Biosciences). Genomic organisation of the hTERT gene and the location of Taqman primer–probe sets are shown in Figure 1. We designed primers and probes to amplify specially only one form of hTERT (Table 1). Primers and probe sets for hTR are also described in Table 1. In order to generate a standard curve, we constructed plasmids that contain each amplified fragment using a pT7Blue T vector-2 kit (Novagen, Darmstadt, Germany). The Taqman *β*-actin kit (Applied Biosystems, Foster City, CA, USA) was also used for normalisation of the amount of cDNA used in each PCR. The resulting cDNA (4 *μ*l) was used in each RT–PCR, and then analysed by a 7000 Sequence Detection System (Applied Biosystems). For Taqman assay, a 50 *μ*l of PCR sample contained Taqman universal master mix (Applied Biosystems, Foster City, CA, USA), 3 pmol of each primer pairs and 5 pmol of the corresponding probes were used as recommended by the manufacturer. The PCR conditions were 95°C for 10 min, followed by 55 cycles of 95°C 10 s and 60°C for 1 min. A serial dilution of plasmids was used in each PCR cycle in separate tubes and served as a standard curve. The amount of gene expression in each sample was then expressed as copy numbers per microgram of RNA with respect to the standard curve.

### Mutation analysis of *hTR*

PCR-direct sequencing was carried out in order to exclude mutation of the *hTR* gene (NT_005612.14). We designed two pairs of primers to detect mutation of the *hTR* gene: hTR-1F (7597157–7598138), 5′-CTCATGGCCGGAAATGGAAC and hTR- 1R (7597633–7597652), 5′-TCTTCCTGCGGCCTGAAAGG; amd hTR-2F (7597864-7597842), 5′-GCCTTCCACCGTTCATTCTAGAG, and hTR-2R (7597413–7597432), 5′-TTTGGAGGTGCCTTCACGTC. The PCR conditions were as follows: preheating at 95°C for 10 min, followed by 40 cycles 95°C for 30 s, 64°C for 30 s and 72°C for 1 min, and a final extension 72°C for 10 min. Reactions for direct sequencing of the PCR product were performed with BigDye Terminator ver3.1 (Perkin-Elmer Cetus, Freemont, CA, USA).

### Statistical analysis

Analysis of variance (one-way ANOVA), correlation analysis, linear regression, Student's *t*-test and the Mann–Whitney *U*-test were calculated using StatView (Brain Power Inc., Calabasas, CA, USA) software for the Macintosh personal computer. Values of *P*<0.05 indicate a statistically significant difference.

## RESULTS

### Validation of quantification system of hTERT, its spliced forms and hTR

Taqman RT–PCR was validated using a plasmid that contained the target sequence of full-length hTERT+*α*+*β*. There was a linear correlation of full-length hTERT+*α*+*β* mRNA between 10^1^ and 10^6^ molecules. Similarly, a linear correlation was observed in each splicing form of hTERT and hTR (data not shown).

### Functionally active telomerase is associated with full-length hTERT expression, but did not correlate with hTR expression

In acute leukaemia cells, the relative telomerase activity measured by TRAP assay is associated with the expression level of full-length hTERT+*α*+*β* mRNA (*P*=0.0024) (Figure 2A). In contrast, there was no correlation between telomerase activity and hTR expression (*P*=0.6753) (Figure 2B). Of note is that there are some exceptional cases showing low telomerase activity despite high copy numbers of hTERT+*α*+*β* (Figure 2A, arrow). We also found two cases of AML showing high telomerase activity with detectable but low copy numbers of hTERT+*α*+*β* (Figure 2A, arrowhead).

There is some overlap between telomerase activity in leukaemia cells and that in normal blood cells; therefore, we arbitrarily separated acute leukaemia patients into two groups according to the relative telomerase activity as reported previously (Ohyashiki *et al*, 1997): one with high telomerase activity, equivalent to immortal cells, relative telomerase value greater than 30 (Group-H), and the other with low to moderate telomerase activity (Group-L). The hTERT expression level is significantly high in Group-H (*P*=0.0013) (Figure 3A), while association between telomerase activity and hTR expression was not significant (Figure 3B). This indicates that functionally active telomerase activity is generally associated with hTERT expression, but in some cases the TERT expression does not simply reflect the enzymatic activity.

### Ratio of hTR and hTERT is critical to determine enzymatic activity of telomerase

To address the question as to why some patients show low telomerase activity despite high hTERT+*α*+*β* expression, we next compared the ratio of hTR and hTERT. The Group-L patients showed significantly lower copy numbers of hTR (*P*=0.0284), and the hTR/hTERT ratio was significantly lower than those in Group-H patients (*P*=0.0094) (Figure 4). This indicates the possibility that the combination of full-length hTERT and hTR is necessary to create a functionally active telomerase activity in leukaemia cells *in vivo*. The quantitative relationships between functionally active telomerase activity and its components are shown in Figure 5. There was an obvious difference between patients with low telomerase activity, despite high full-length hTERT expression (UPN41, 40 and 44, Figure 5A–C, respectively) and patients with high telomerase activity (UPN15, Figure 5D). We next analysed the mutation of the *hTR* gene in three patients showing a marked discrepancy between hTERT+*α*+*β* expression and telomerase activity, in order to determine whether this phenomenon is related to mutation of *hTR*. No case showed mutation of *hTR* gene within the limit of our primers. This indicates that the discrepancy between expression of full-length hTERT and functionally active telomerase activity is possibly due to the quantity of hTR but not to the gene structure of *hTR*.

### Role of nonactive splicing forms of hTERT

To clarify whether the splicing mechanism of hTERT really affects the level of functional telomerase activity or not, we next compared the expression level of hTERT+*α*+*β* and three spliced forms of hTERT. The expression level of full-length hTERT+*α*+*β* mRNA was generally associated with levels of spliced variants hTERT+*α*–*β* (*P*=0.0434) (Figure 6B) and hTERT−*α*−*β* (*P*=0.0084) (Figure 6C), while the relationship between the expression level of full-length hTERT+*α*+*β* mRNA and those of spliced variant hTERT−*α*+*β* was not statistically significant (*P*=0.1109) (Figure 6A). The ratio of spliced form/full-length hTERT+*α*+*β* mRNA varied, but tended to be higher in Group-L patients compared to those in Group-H, although the difference was not always statistically significant: hTERT+*α*−*β*/full-length hTERT+*α*+*β* (*P*=0.101), hTERT−*α*+*β*/full-length hTERT+*α*+*β* (*P*=0.048) (Figure 6D) and hTERT−*α*−*β*/full-length hTERT+*α*+*β* (*P*=0.201). This indicates that increase of nonfunctional splicing form of hTERT may play some role in telomerase downregulation.

## DISCUSSION

Telomerase and telomere length are two important markers that are rapidly gaining importance as targets for cures of several age-related diseases including cancer. We therefore sought to determine whether therapeutic approaches to leukaemia targeting telomerase should consider the quantitative relationship between telomerase and its components or not. Acute leukaemia is composed of a heterogeneous population in terms of cell lineage, cell differentiation and proliferative potential. In the current study, the level of telomerase activity and telomerase components revealed considerable patient-to-patient variation; however, we found telomerase activity is significantly associated with hTERT expression in most patients but did not correlate with hTR expression. We also found that in some cases telomerase activity was low, despite high copy numbers of full-length hTERT mRNA correlating with low copy numbers of hTR. This is of particular interest given that hTR has now been shown to be limiting for telomere homeostasis *in vivo*, as seen in DKC (Mitchell *et al*, 1999; Vulliamy *et al*, 2001).

Recently, mutations of *hTR* have been reported in a subset of aplastic anaemia (Vulliamy *et al*, 2002). Although it is still controversial whether the genetic change of *hTR* sequence is polymorphism or not (Wilson *et al*, 2003; Yamaguchi *et al*, 2003), Ly *et al* (2003) demonstrated that naturally occurring *hTR* sequence mutation polymorphism in such patients can inhibit telomerase activity by disrupting critical structures within the *hTR* core domain. Unlike DKC, neither mutation nor deletion of *hTR* was detected in this study by direct sequencing. This suggests that the amount of hTR is so low that as a result there is an excess of unbound hTERT mRNA. Indeed, the expression level of hTR is consistent in leukaemia cell lines showing high telomerase activity (Yi *et al*, 2001). The mechanism of telomerase regulation in acute leukaemia cell is likely to be different from those in DKC and bone marrow failure syndrome; however, the ratio of hTR and hTERT might play an important role to contribute functionally active telomerase activity and telomere homeostasis *in vivo*, whether or not mutated *hTR* affect telomerase activity via haploinsufficiency.

In the current study, we found two exceptional cases with high telomerase activity despite low expression of hTERT; therefore, we could not completely rule out the possibility that hTERT-associated proteins such as heat-shock proteins may affect the activity of the telomerase holoenzyme.

Alternative splicing machinery of hTERT is considered to be tissue specific and to influence telomere lengths during human development (Ulaner *et al*, 2001). It has been shown that hTERT RNA alternative splicing mediates telomerase downregulation induced by the G-quadruplex ligand 12459 (Gomez *et al*, 2004). However, the ratios of spliced nonactive forms and full-length hTERT in primary acute leukaemia cells are highly varied. Of note is that the ratio of splicing variants and full-length hTERT is lower in patients with high telomerase activity (*n*=7) than that in patients without high telomerase activity (*n*=31). It is known that splicing variants lack the *α* site function as a dominant-negative inhibitor of telomerase (Colgin *et al*, 2000; Yi *et al*, 2001). Although we could not show direct evidence that the spliced inactive variant of hTERT downregulates full-length wild-type hTERT, it is likely that splicing variant mRNA is related with some regulatory mechanism in acute leukaemia cells without exhibiting high telomerase activity. While, the meaning of these epiphenomena is still uncertain, the regulatory mechanism of telomerase in leukaemia cells with low telomerase activity appears to be similar to that in normal counter parts. Zaffaroni *et al* (2002) reported that alternative splicing mechanisms of hTERT that regulate telomerase activity in normal tissue might be lost during malignant transformation in breast tumours. Taken together with Zaffaroni's observation (2002), our results suggest that acute leukaemia cells with high telomerase activity might lose their regulatory mechanism during disease progression.

Our findings suggest that the regulatory mechanisms in leukaemia cells may be heterogeneous; therefore, the therapeutic approach targeting telomerase should be considered based on the quantitative relationship between telomerase and its components. While the number of patients studied in the current study is limited, our results suggest the necessity, and provide the basis, for more detailed studies on the complex regulatory mechanism of telomerase activity in haematologic neoplasia that may lead to the development of new cancer therapeutic strategies.

## Figures and Tables

**Figure 1:** The genomic organisation of the *hTERT* gene and the location of Taqman primer–probe sets. To quantify potentially active full-length hTERT (+*α*+*β*), we used an ex6-F primer and ex7-R primer. We used an *α*-del-F primer and ex7-R primer for a spliced variant of hTERT−*α*+*β*, and an ex-6F primer and *β*-del-R primer for the spliced variant of hTERT+*α*−*β*, and an *α*-del-F primer and *β*-del-R primer for hTERT−*α*−*β*. For all types of hTERT mRNA, we uniformly used an ex6 probe. The *α* site causes a 30-base deletion resulting in a no-frameshift mutation, and the *β* splice site results in a 182-base deletion resulting in a nonsense mutation. The size of the PCR product produced by each primer set depends upon the alternative splicing of the hTERT transcript in the sample.

**Figure 2:** Relationship between telomerase activity level and hTERT+*α*+*β* mRNA expression level (**A**) and telomerase activity level and hTR RNA expression level (**B**). The level of telomerase activity was generally associated with the copy numbers of full-length hTERT mRNA, but there were some exceptional cases showing low telomerase activity despite high copy numbers of hTERT+*α*+*β* (arrow) and cases showing high telomerase activity with detectable but low copy numbers of hTERT+*α*+*β* (arrowhead).

**Figure 3:** Expression level of hTERT (**A**) and hTR (**B**) in acute leukaemia patients. Group-H: Patients with high telomerase activity; group-L: patients with low–moderate telomerase activity. Expression level of hTERT is significantly higher in Group-H, but there was no difference of hTR expression level in the two groups.

**Figure 4:** Expression level of hTR in patients with high hTERT mRNA expression. Group-H: Patients with high telomerase activity; group-L: patients with low–moderate telomerase activity. The expression level of hTR is significantly lower in Group-L.

**Figure 5:** The quantitative relationship between functionally active telomerase activity and its components. Shapes of three elements (full-length hTERT, hTR and relative telomerase activity) are different in patients with low telomerase activity despite high full-length hTERT expression (**A**–**C**) and that in a patient with high telomerase activity (**D**).

**Figure 6:** Relationship between hTERT+*α*+*β* mRNA expression level and its spliced forms (**A**: hTERT−*α*+*β* (**B**) hTERT+*α*−*β* (**C**) hTERT−*α*−*β*). The ratio of hTERT−*α*+*β*/hTERT+*α*+*β* mRNA (full-length hTERT) is significantly lower in Group-H (**D**) (*P*=0.048).

**Table 1:** Primers and probes for quantification of the hTERT mRNA and hTR RNA

*hTERT*	
Ex5, 6-F primer	5′- GAG CTG TAC TTT GTC AAG GTG GGA TG-3′
*α*-Del-F primer	5′- CTG AGC TGT ACT TTG TCA AGG ACA GG-3′
Ex7-R primer	5′- GGC TGG AGG TCT GTC AAG GTA GAG A-3′
*β*-Del-R primer	5′- GCA CTG GAC GTA GGA CGT GGC T-3′
Ex6 probe	5′- FAM-CAACCCCAGAACACGTACTGCGTGCGT-3′
	
*hTR*	
hTR-F primer	5′- CGC TGT TTT TCT CGC TGA CTT-3′
hTR-R primer	5′- TGC TCT AGA ATG AAG GGT GGA A-3′
hTR probe	5′-FAM-CAG CGG GCG GAA GGA CCT CG-3′

hTR=human telomerase template RNA; FAM=5-carboxyfluorescein; hTERT= human telomerase reverse transcriptase.

To generate full-length hTERT+*α*+*β*, ex5, 6-F primer and ex-7-R primer were used. To generate splicing forms of hTERT, we used the following primer sets: hTERT+*α*−*β*; ex5, 6-F and *α*-del-R primers, hTERT−*α*+*β*; *α*-del-F and ex7-R primers, hTERT−*α*−*β*; *α*-del-F and *β*-del-R primers. The ex6 probe was used to detect full-lengh hTERT+*α*+*β* as well as splicing forms of hTERT.
